The article "Salvage Radiosurgery for Selected Patients with Recurrent Malignant Gliomas" was published in 2014. Journal: Biomed Res Int.

# Salvage Radiosurgery for Selected Patients with Recurrent Malignant Gliomas

**DOI:** 10.1155/2014/657953

**Published:** 2014-05-07

**Authors:** Miguel Martínez-Carrillo, Isabel Tovar-Martín, Mercedes Zurita-Herrera, Rosario Del Moral-Ávila, Rosario Guerrero-Tejada, Enrique Saura-Rojas, Juan Luis Osorio-Ceballos, Juan Pedro Arrebola-Moreno, José Expósito-Hernández

**Affiliations:** ^1^Radiation Oncology Department, Virgen de las Nieves University Hospital, 18014 Granada, Spain; ^2^Neurosurgery Department, Virgen de las Nieves University Hospital, 18014 Granada, Spain; ^3^Medical Physics Department, Virgen de las Nieves University Hospital, 18014 Granada, Spain

## Abstract

*Purpose*. To analyse the survival after salvage radiosurgery and to identify prognostic factors. *Methods*. We retrospectively reviewed 87 consecutive patients, with recurrent high-grade glioma, that underwent stereotactic radiosurgery between 1997 and 2010. We evaluated the survival after initial diagnosis and after reirradiation. The prognostic factors were analysed by bivariate and multivariate Cox regression model. *Results*. The median age was 48 years old. The primary histology included anaplastic astrocytoma (47%) and glioblastoma (53%). A margin dose of 18 Gy was administered in the majority of cases (74%). The median survival after initial diagnosis was 21 months (39 months for anaplastic astrocytoma and 18.5 months for glioblastoma) and after reirradiation it was 10 months (17 months for anaplastic astrocytoma and 7.5 months for glioblastoma). In the bivariate analyses, the prognostic factors significantly associated with survival after reirradiation were age, tumour and treatment volume at recurrence, recursive partitioning analyses classification, Karnofsky performance score, histology, and margin to the planning target volume. Only the last four showed significant association in the multivariate analyses. *Conclusion*. stereotactic radiosurgery is a safe and may be an effective treatment option for selected patients diagnosed with recurrent high-grade glioma. The identified prognostic factors could help individualise the treatment.

## 1. Introduction

Gliomas are primary malignant brain tumours that arise from glial cells. The World Health Organization (WHO) has classified gliomas into four grades of ascending malignancy [1]. According to this classification, grade III and grade IV, also known as anaplastic astrocytoma (AA) and glioblastoma multiforme (GBM), respectively, are the most aggressive and are termed high-grade gliomas (HGG) [1]. The current standard treatment for glioblastoma patients includes maximal surgical resection, followed by temozolomide (TMZ) concomitant with external beam radiation (EBRT), and then subsequently with additional TMZ cycles, following the Stupp protocol [2]. Despite significant improvements in neuroimaging, surgical techniques, radiotherapy, and chemotherapy, the prognosis for these patients is still poor, with a median survival of 14.6 months and an overall survival of 27% after 2 years, dropping then to under 10% after 5 years [2].

The article "Salvage Radiosurgery for Selected Patients with Recurrent Malignant Gliomas" was published in 2014. Journal: Biomed Res Int.

Recurrence occurs in more than 90% of the patients [3] and its treatment is not clearly established with a median survival of 3–6 months without treatment [4]. Different options of treatment include: repetition of surgical resection, reirradiation with EBRT, brachytherapy or stereotactic radiosurgery (SRS), chemotherapy, novel therapies, or a combination of the above. Due to the highly invasive nature of HGG and the subsequent difficulty to delineate it, local treatment does not seem to make sense. However, the majority of treatment failures are within the irradiated field; up to 90% of recurrences occurred within 2 cm of the tumour margins [5]. For this reason, local control is one of the main goals of the treatment of recurrent HGG.

Tumour resection is a good option for salvage treatment, but it is associated with many postoperative complications. EBRT exposes the brain to a high risk of radiation-related toxicity and necrosis. Brachytherapy is also associated with serious side effects like infections or risk of haemorrhage. All of this suggests a potential key role for SRS in the management of recurrent HGG; in addition, these tumours are relatively hypoxic with low *α*/*β* and a priori good responders to hypofractionated irradiation [4–6].

First conceived by Lars Leksell in 1951, stereotactic radiosurgery (SRS) is an irradiation modality that combines stereotactic technique with highly focused high-energy radiation treatments, making it possible to deliver large doses of radiation to an extremely small target [7].

The experience of reirradiation with radiosurgery for recurrent HGG is limited. At our institution, we have performed single fraction reirradiation (SRS) in selected patients with relatively well defined recurrent tumors as seen on imaging studies, which have an adequate volume.

In this study, we investigated our clinical data to evaluate the efficacy of SRS as a salvage treatment and the potential prolongation of survival time in 87 patients. Additionally we reported the results of overall and post-SRS survival and prognostic factors in patients with recurrent HGG treated with linear accelerator- (LINAC-) based radiosurgery over a 12-year period.

## 2. Patients and Methods

### 2.1. Patients

Between 1997 and 2010, 87 consecutive adult patients were treated at Virgen de las Nieves University Hospital (Granada, Spain). All of them underwent SRS LINAC as salvage treatment for recurrent HGG with the following features: (1) pathologically confirmed diagnosis of AA or GBM at the time of initial management; (2) underwent subsequent fractionated radiotherapy treatment with radical intent; (3) developed new or increasing contrast-enhanced lesions at the margin of primary localization in the follow-up magnetic resonance imaging (MRI) after radiotherapy, indicating tumour recurrence or progression; and (4) the size of the lesion was <3 cm.

The article "Salvage Radiosurgery for Selected Patients with Recurrent Malignant Gliomas" was published in 2014. Journal: Biomed Res Int.

Data were retrospectively collected by reviewing medical records, last followup in the hospital, and MRI studies and contacting patients and/or families. This way, we obtained information about age, gender, recursive partitioning analyses (RPA) classification [8], Karnofsky performance status (KPS) score, histology as World Health Organization (WHO) grade 3 gliomas AA or GBM, time to relapse, tumour and treatment volume at recurrence, margin to the planning target volume, dose administered, and radiological and neurological responses. Dates of death were obtained from National Death Index (INDEF, Spanish initials).

### 2.2. Radiosurgery

Outpatient radiosurgery was indicated by a medical staff composed of neurosurgeons, radiologists, radiation oncologists, and physicists involved in treatment planning and target volume determination for all patients.

Treatment was planned on the image fusion of computed tomography (CT) and MRI data, for the contrast-enhancing regions on T1-weighted MRI images, and was delivered using a linear accelerator (LINAC) (Varian 2100) equipped with micro-multileaf collimators (MMC) using 6 MV photons. A BrainLAB stereotactic head frame (BrainLAB A.G., Heimstetten, Germany) was used for every patient. BrainLAB cones were used for the treatment until 2004 when dynamic micro-multileaf collimator was incorporated (Figure 1).

The prescribed dose for reirradiation was based on tumour volume, prior radiation dose, time since EBRT, and location of the lesion with proximity to eloquent brain or radiosensitive structures. The GTV (contrast-enhancing lesion in T1-weighted MR images) was expanded by 0–6 mm to generate the planning target volume (PTV). This expansion was related to the year of treatment (without any expansion during the first five years), in the size and location of the recurrence.

### 2.3. Followup

After SRS, patients were seen for a follow-up visit after 8 weeks and thereafter in 3 months intervals. Each follow-up appointment consisted of a thorough clinical examination, including a neurological assessment and a contrast-enhanced MRI. Local control (LC) was defined as stabilization or decrease of lesion size or enhancement on imaging and lack of consistently increased surrounding T2 signal changes on serial examinations. Local failure was defined as persistent increase in size of the contrast-enhancing lesion (>20% volume increase) or new contiguous areas at the margin of treatment and concomitant T2 signal change. Toxicity was also collected. Differentiating second-time recurrence tumour after SRS from radiation injury based on MRI is difficult. Progressive contrast enhancements over time may represent either a mixture of a viable tumour and radiation-induced necrosis or radiation injury only. Metabolic imaging, MR spectroscopy, and MR perfusion were used as supplements in some uncertain cases.

The article "Salvage Radiosurgery for Selected Patients with Recurrent Malignant Gliomas" was published in 2014. Journal: Biomed Res Int.

### 2.4. Statistical Analyses

The aim of these studies is to examine the overall survival, post-SRS survival, and the identification of prognostic factors with influence on survival after SRS.

Overall survival was calculated from the time of the primary diagnosis to the time of death or last followup. Survival after SRS was calculated from the time of SRS until the death of last followup, using the Kaplan-Meier method.

Bivariate statistical analyses were performed to examine the relationships between the duration of survival after SRS and different variables at the time of the treatment, using Cox regression models. In a first step, those variables which were statistically significant in the bivariate analyses were included in the multivariate model that was finally built using a backward stepwise technique. Diagnosis of the models was performed in order to ensure the goodness of the fit and the fulfilment of implementation conditions. Hazard ratios (HRs) with 95% confidence intervals (CIs) were calculated. Two-sided* P* values less than 0.05 were considered significant. SPSS version 12 (SPSS, Chicago, IL) was used for statistical analyses, except for multivariate analyses that were performed by “R” version 3.0.2.

## 3. Results

### 3.1. Patients

The initial treatment characteristics are shown in Table 1. This initial treatment included: surgery, EBRT within 8–12 weeks after surgery with doses varying 54–66 Gy (mean 60 Gy), and adjuvant chemotherapy in 63 patients. Surgery with complete resection was performed in 43 patients (49.4%). From 1999 up to and including 2004, patients received EBRT alone or in combination with procarbazine, lomustine, and vincristine (PCV). From 2005, patients received the Stupp protocol [9] with temozolomide and EBRT, except for patients without good medical conditions who underwent exclusive EBRT. Thus, 51 patients (58.6%) were treated with the Stupp protocol, 12 patients (13.8%) were treated with EBRT in combination with PCV, and 24 patients (27.6%) were treated with EBRT alone.

The article "Salvage Radiosurgery for Selected Patients with Recurrent Malignant Gliomas" was published in 2014. Journal: Biomed Res Int.

Clinical features in recurrence are summarised in Table 2. Out of 87 patients, 43 were males and 44 females; median age was 49 years old; 41 patients with anaplastic astrocytoma (AA) and 46 with glioblastoma (GBM). The diagnosis was histologically confirmed in all patients. KPS score was higher than 80 in 40 patients. 51 patients (29 with AA and 20 with GBM) had surgery for the first recurrence and radiosurgery for the residual tumour seen on the postoperative MRI after reoperation or for a second recurrence. The median time interval from diagnosis to SRS treatment was 13.8 months (range 5–61 m).

### 3.2. Radiosurgery and Radiological and Clinical Responses

The median prescribed dose was 18 Gy (range 14–20). The median tumor volume and PTV volume were 4 cc and 6 cc, respectively. The margin of the GTV to create the PTV was 0 mm in the majority of treatments (48.3%) followed by 5 (20.7%). The treatment was administered by cones in 40.2% of cases and by MMC in 59.8%. The majority of patients received only one SRS treatment (89%), while the remainder underwent more than one course of SRS (9.8% two SRSs and 1.2% three SRSs).

The median follow-up after SRS was 10 months (range 1–141 months). The initial radiological response was complete in 7.8%, partial in 24.7%, stabilisation in 32.5%, and progression in 26%. In 9% of the patients the response could not be evaluated, because of death before the MRI. These patients are considered as nonresponders. At the initial evaluation after the SRS, 17.1% of patients were clinically better than before the treatment, 32.9% remained without change, 21.4% were neurologically worse, and 28.6% were not evaluated because of death before the first follow-up visit or incomplete data in the clinical record.

There were no cases of treatment-related adverse events or episodes of acute neurological toxicity. On the follow-up images (10%) there was an increasing oedema with a transient worsening of neurological function for the patients; all of this was considered as adverse radiation effects.

The treatment of local failure post-SRS consisted of surgical resection in three patients, changes in chemotherapy regimen in five patients, and no further treatment for the remainder.

### 3.3. Survival and Prognostic Factors

At the end of the study 7 patients (8%) were alive with no evidence of disease, 5 patients (5.7%) were alive with disease, and 75 patients (86.2%) were dead. The cause of death was the progression of the tumour in all patients.

Table 3 shows the information about survival. The median overall survival was 21 months (range 9–151 months), although patients treated by Stupp protocol had higher survival than patients treated by other treatments [10]. Initial treatment (Stupp versus others) was not significantly associated with overall survival (HR = 0.79; 95 % CI = 0.49–1.25). The actuarial global survival rates after 12, 24, and 36 months were 88.5%, 46%, and 35.6%, respectively (Figure 2(a)). The median survival after SRS was 10 months (range 1–141 months), 7.5 months for GBM (range 1–140), and 17 months for AA (4–141). The actuarial survival after SRS rate was 37.9% after 12 months, 28.7% after 24 months, and 25.3% after 36 months (Figure 2(b)).

The article "Salvage Radiosurgery for Selected Patients with Recurrent Malignant Gliomas" was published in 2014. Journal: Biomed Res Int.

The variables included in the analyses of the prognostic factors of post-SRS survival were age (year old), gender, KPS score, RPA classification, histology (AA or GBM), initial surgery (complete or not), initial treatment (Stupp protocol versus other treatments), time of recurrence (months), focality (unifocal or multifocal), tumour volume (cubic centimeter), treatment volume (cubic centimeter), margin to the PTV (millimeter), and dose (Gy) administered. In the bivariate analyses (Table 4) the following variables were significantly associated with survival post-SRS: age (years old) (HR = 1.04; 95% CI = 1.01–1.05), KPS ≤ 80 versus > 80 (HR = 2.59; 95% CI = 1.55–4.3), RPA IV versus III (HR = 2.39; 95% CI = 1.18–4.82), RPA V versus III (HR = 6.32; 95% CI = 2.82–14.14), GBM versus AA (HR = 2.45; 95% CI = 1.53–3.94), tumour volume (cubic centimetre) (HR = 1.04; 95% CI = 1.01–1.07), treatment volume (cubic centimetre) (HR = 1.03; 95% CI = 1.01–1.06), and margin to the PTV (millimetre) (HR = 0.77; 95% CI = 0.67–0.87). In the multivariate analyses (Table 3) we found that the risk of sudden death was 2.08 times higher in KPS ≤ 80 than KPS > 80 (95% CI = 0.28–0.83) (Figure 3(a)), 3.13 times higher in GBM than AA (95% CI = 1.79–5.48) (Figure 3(b)), 3.46 times higher in RPA IV than RPA III (95% CI = 1.61–7.46), 7.29 times higher in RPA V than RPA III (95% CI = 3.23–16.34) (Figure 3(c)), and 3.19 times higher in PTV margin 0 than PTV ≥ 1 (95 % CI = 1.91–5.31).

## 4. Discussion

Poor prognosis of this HGG with high risk of relapse, mainly within 2 cm of the resection cavity, suggests there is a need to improve local treatment [4]. Hau et al. [11] compared patients who were treated with aggressive salvage therapy including SRS with a group of patients who received no salvage treatment. In that study, the median actuarial survival after recurrence was 8.2 months in the intervention group and 2.2 months in the nonintervention group, indicating that salvage treatment was beneficial.

Several authors have studied the optimal moment to administer SRS: as an initial treatment or as an adjuvant treatment for recurrence [6, 12]. Nowadays, the study with the highest level of evidence is Radiation Therapy Oncology Group 93-05 [12]. Although it was highly criticised, the conclusion was that the addition of SRS at the time of initial treatment did not appreciably enhance survival, quality of life, or neurocognition for GBM. However, Kong et al. [13] showed a survival benefit of SRS as salvage treatment compared with historic control. So far, the main role of SRS takes place at the time of recurrence, for this reason, our department does not recommend SRS as initial treatment.

The article "Salvage Radiosurgery for Selected Patients with Recurrent Malignant Gliomas" was published in 2014. Journal: Biomed Res Int.

Managing recurrent HGG is particularly challenging. Surgery is well established as newly diagnoses HGG; however, the reoperation has a low median postoperative survival and high complication rates due to the infiltrative growth pattern of gliomas [14–16]. Skeie et al. [17] reviewed patients treated with SRS, surgery, or both. For recurrent GBM the median survival for SRS was significantly better than surgery. Surgery could be used to decrease the size of a large tumour before SRS. This way, 59% of our patients underwent surgery as salvage treatment after recurrence that allowed the treatment with SRS for the residual tumour. EBRT increases the risk of late cumulative radiation injury, although the recent advances in radiotherapy that reduce the radiation to surrounding brain tissue can turn this treatment into a useful option for tumours with a larger volume [4]. Brachytherapy can have side effects as radiation necrosis, hemorrhage, and infection [4]. Thus, there is a clear advantage of SRS over brachytherapy: the noninvasive approach. There have been many studies suggesting that SRS is effective mainly for HGG [13, 18–20].

Related to adverse side effects due to reirradiation by SRS, early toxicity as headache, nausea, vomiting, and so forth is medically managed, while late complication involves radiation necrosis that typically develops one to three years after radiation. The incidence reported by the literature varies from 0% [21, 22] to 30% [23, 24] and is associated with tumour volume [24]. In our series, none of the patients had radiation necrosis, probably given the short life expectancy. In addition, we believe that SRS provides a highly precise delivery of radiation dose sufficient to induce tumour cell death while sparing surrounding host tissue. For this reason, we think reirradiation by SRS is safe for small tumours.

We analysed our series with 87 patients treated with SRS at the moment of the recurrence. We used a LINAC equipped with micro-multileaf collimators (MMC) using 6 MV photons and a BrainLAB stereotactic head frame. There are different SRS modalities (LINAC, Cyberknife and Gamma knife), and most of the published articles describe the experience with Gamma Knife. However, there is no evidence of which modality is better. The majority of patients received 18 Gy in one fraction, and as other authors pointed, because of the high radiation dose already given in the initial treatment with EBRT, it is difficult to administer a high dose [17]. Skeie et al. [17] did not find any difference in survival when they compared patients who received more than 12 Gy versus ≤12 Gy. In addition, the dose administered was not correlated to survival post-SRS in our study.

The article "Salvage Radiosurgery for Selected Patients with Recurrent Malignant Gliomas" was published in 2014. Journal: Biomed Res Int.

The median overall and post-SRS survival in our study is in accordance with the literature (Table 5). The median post-SRS survival varies between 6.5 months [25] and 26 months [13]. These differences may be due to the inhomogeneity among the studies (clinical features of the patients, histological type, modalities of treatment after SRS, and so forth). The study with the largest number of patients is Kong et al.'s study [13] with a post-SRS survival of 26 months for grade III gliomas and 13 months for grade IV gliomas, different data as RPA classifications were not reported.

Favourable prognostic factors derived from the most relevant studies published (Table 5) include higher prescription dose, adequate SRS margin, anaplastic astrocytoma, smaller tumour volume, younger age, higher KPS, better RPA, location in noneloquent area, unifocality, and concurrent chemotherapy. However, among the different prognosis factors analysed in the present study, only KPS score, RPA, histology, and margin to the PTV made statistically a significant influence on post-SRS survival in the multivariate analyses. The identification of prognostic factors varies among studies. The difference may be due, in part, to the definition and/or adherence of eligibility criteria, clinical features of the patients, characteristic of the treatment, and so on. Other molecular prognosis factors as O-6-methylguanine-DNA methyltransferase (MGMT) methylation, 1p/19q deletion, or isocitrate dehydrogenase 1/2 (IDH1/2) mutation [26] were not included in these studies, probably because the role of this molecular factors is fairly recent.

Shrieve et al. [27] showed that while under 40 years old patients had a median survival of 49 months; over 40 years old patients had a median survival of 18.2 months (*P* < 0.001). In our study the age was associated with the post-SRS survival only in the bivariate analyses; thus, for each extra year of life the risk of sudden death was multiplied by 1.04 (95% CI = 1.01–1.05). We did not find this correlation in the multivariate analyses, perhaps because the variability explained by this variable in the bivariate analyses was later explained by the RPA classification in the multivariate model.

The article "Salvage Radiosurgery for Selected Patients with Recurrent Malignant Gliomas" was published in 2014. Journal: Biomed Res Int.

The tumour and treatment volumes were identified as prognosis factor for the post-SRS survival in the bivariate analyses but not in the multivariate analyses. Kong et al. [13] and Combs et al. [28] obtained the similar results, although the latter treated patients with fractionated stereotactic radiotherapy instead of SRS.

According to our statistical analyses, higher KPS score was statistically significant correlated with post-SRS survival. In our study the cut-off point was KPS score of 80 (Figure 2(a)), while Cuneo et al. [29] reported the same correlation but with a cut-off point of 70 in the KPS score. Other authors have shown KPS score as prognosis factor for survival with a cut-off point of 90 [22, 24].

RPA classification was a significant predictive value of survival on bivariate and multivariate analyses in this series, reinforcing the predictive value of the RPA classification even with salvage treatments. A survival benefit from SRS for patients with class III through V has also been suggested by Ulm et al. [30] and Skeie et al. [17].

We found that the risk of sudden death was 3.13 times higher in GBM than AA (95% CI = 1.79–5.48) (Figure 2(b)). In HGG group, grade III presents a significant favourable prognosis with respect to grade IV, for overall and postsalvage SRS survival. Larson et al. [31] found that the post-SRS survival was 68 weeks and 38 weeks for grade III and grade IV gliomas, respectively. Kong et al. [13] found similar results with post-SRS survival of 26 months and 13 months for grades III and IV, respectively.

PTV margin was a statistical significant protective factor. Several authors defend the use of an “extended field” to cover the potential microscopic expansion [32, 33]. As mentioned above, this strategy is supported by the acknowledgment that this kind of tumours tend to progress within 2 cm of the contrast-enhancing edge. Koga et al. [32] found a statistically significant difference in the local control between conventional SRS (47%) and extended field (93%). However, the “extended field” depends on the tumour volume, location,and if there are close organs at risk, considering that in reirradiation the treatment volume has a strong correlation with the toxicity.

To obtain better results for this kind of tumours, different strategies are mentioned:

- Imaging to improve the target delineation and to evaluate the results after treatment.
- New chemotherapy agents and targeted therapies as bevacizumab [29].
- Molecular characterisation of these tumours as the determination of the methylation status of MGMT [26].

The article "Salvage Radiosurgery for Selected Patients with Recurrent Malignant Gliomas" was published in 2014. Journal: Biomed Res Int.

The main weakness of our study is the retrospective character of the study with a heterogeneous population and nonuniform treatment modalities and selection bias because patients who are candidates for salvage SRS treatment tend to have more favourable prognosis factors than those ineligible patients. However, due to the low incidence of these tumours, a prospective study is difficult and in clinical practice, patients diagnosed with this entity are not homogeneous and neither is the initial treatment which depends on the medical condition of the patients. You can find the same problem related to the homogeneity of the sample in other published articles [3, 4, 13]. In addition, our series has a large number of patients and the results are in accordance with the literature.

## 5. Conclusion

There is no class I evidence establishing a “standard of care” for recurrence. Because local recurrence remains the predominant pattern of failure in patients with HGGs, local salvage treatment with SRS is appropriate and safe and may contribute to a prolonged survival in young patients with AA histology who have a good KPS score and RPA classification, a small volume, and are treated with an adequate margin. In addition, it seems multimodality treatment is better than no salvage therapy, for this reason, we recommend second surgery to reduce the volume of the recurrence and to complete the treatment with SRS if possible.

## Figures and Tables

**Figure 1:** An example of radiosurgery treatment in our department.

**Figure 2:** Overall and post-SRS survival. Kaplan-Meier survival function.

**Figure 3:** Prognosis factors, Kaplan-Meier survival function.

**Table 1:** Initial treatment features.

Parameters	Number of patients (%)
Number or patients	87
Primary surgery Complete resection Subtotal resection Biopsy	43 (49.4) 23 (26.4) 21 (24.2)
Adjuvant therapy Stupp protocol PCV + EBRT EBRT without chemotherapy	51 (58.6) 12 (13.8) 24 (27.6)

**Table 2:** Patient treatment characteristics at recurrence.

Parameters	Number of patients	Patients treated by Stupp protocol	Patients diagnosed with AA	Patients diagnosed with GBM
Numbers of patients	87	51	41	46
Gender Male Female	43 (49.4%) 44 (50.6%)	27 (52.9%) 24 (47.1%)	16 (39%) 25 (61%)	27 (58.7%) 19 (41.3%)
Age (years) median (range)	48.7 (18–78)	47 (26–71)	45 (18–78)	49.5 (26–78)
KPS Mean (range) KPS > 80 KPS ≤ 80	83 (60–100) 40 (46%) 47 (50%)	90 (70–100) 28 (54.9%) 23 (45.1%)	90 (70–100) 22 (53.7%) 19 (46.3%)	80 (70–100) 18 (39.1%) 28 (60.9%)
RPA Mean (range)	4.1 (3–5)	4 (3–5)	4 (3–5)	4 (3–5)
Histology Anaplastic astrocytoma Glioblastoma	41 (47.1%) 46 (52.9%)	25 (49%) 26 (51%)	100% 0	0 100%
Time to recurrence (months) Mean (range) ≤8 months 9–12 months >12 months	13.8 (4–61) 29 (33.3%) 30 (34.5%) 28 (32.2%)	11 (4–61) 14 (27.4%) 19 (27.3%) 18 (35.3%)	10 (4–61) 12 (29.3%) 15 (36.6%) 14 (34.1%)	10 (5–28) 17 (36.9%) 15 (32.6%) 13 (30.5%)
Tumour volume (cc) Mean (range) <3 cc 4–7 cc >7 cc	8.7 (1–42.6) 29 (33.3%) 26 (29.9%) 32 (36.8%)	4 (0.36–34.1) 16 (31.4%) 22 (43.1%) 13 (25.5%)	5.2 (1–28) 12 (29.3%) 12 (29.3%) 17 (41.4%)	4 (0.05–34.1) 17 (37%) 14 (30.4%) 15 (32.6%)
Location Unifocal Multifocal	79 (90.8%) 8 (9.2%)	45 (88.2%) 6 (11.8%)	39 (95.1%) 2 (4.9%)	40 (87%) 6 (13%)
Dose radiosurgery Mean (range) Dose ≥ 18 Gy	18.01 Gy (14–20) 76 (87%)	18 Gy (16–20) 46 (90.2%)	18 (15–20) 35 (85.4%)	18 Gy (14–20) 41 (89.1%)
PTV margin Mean (range) 0 mm 1–3 mm >3 mm	1.67 mm (0–6) 43 (49.4%) 22 (25.3%) 22 (25.3%)	2 mm (0–6) 20 (39.2%) 10 (19.6%) 21 (41.2%)	2 mm (0–5) 19 (46.3%) 12 (29.3%) 10 (24.4%)	0 mm (0–6) 24 (52.2%) 10 (21.7%) 12 (26.1%)

The article "Salvage Radiosurgery for Selected Patients with Recurrent Malignant Gliomas" was published in 2014. Journal: Biomed Res Int.

**Table 3:** Survival.

	Stupp protocol	Others Treatments	AA	GBM
OS (median)	21 months	19 months	39 months	18.5 months
Actuarial Sv 12 m 24 m 36 m	88.5% 46% 35.6%	88.9% 36.1% 25%	95.1% 41.5% 30.9%	82.6% 50% 21.7%
Post-SRS Sv	10 months	9 months	17 months	7.5 months
Actuarial post-SRS Sv 12 m 24 m 36 m	37.9% 28.7% 25.3%	30.6% 19.4% 16.7%	70.7% 41.5% 25.7%	30.4% 13% 10.9%

OS: overall survival and Sv: survival.

**Table 4:** Prognostic factors.

Variables	Bivariate analyses		Multivariate analyses	
	HR (95% CI)	*P* value	HR (95% CI)	*P* value
Age	1.04 (1.01–1.05)	*P* < 0.001	Not significant	
KPS (≤80 versus >80)	2.59 (1.55–4.3)	*P* < 0.001	2.08 (0.28–0.83)	*P* = 0.008
RPA				
IV versus III	2.39 (1.18–4.82)	*P* = 0.015	3.46 (1.61–7.46)	*P* = 0.001
V versus III	6.32 (2.82–14.14)	*P* < 0.001	7.29 (3.23–16.34)	*P* < 0.001
Histology (GBM versus AA)	2.45 (1.53–3.94)	*P* < 0.001	3.13 (1.79–5.48)	*P* < 0.001
Tumour volume	1.04 (1.01–1.07)	*P* = 0.005	Not significant	
Treatment volume	1.03 (1.01–1.06)	*P* = 0.013	∗	
Margin to PTV				
0 versus ≥1	0.77 (0.67–0.87)	*P* < 0.001	3.19 (1.91–5.31)	*P* < 0.001

*This variable was not considered for the multivariate analyses because of the strong correlation (0.97 Spearman' s correlation coefficient) with tumour volume.

**Table 5:** Studies of SRS as treatment for recurrent high-grade gliomas.

Study	*N*	Histological grade	Median dose (Gy)	Median volume (cm^3^)	Median post-SRS survival (months)	Prognostic factors
Chamberlain et al., 1994 [34]	15	IV	13.4	17	8	NR
Hall et al., 1995 [35]	25	III–IV	20	28	6.5	Age, KPS
Shrieve et al., 1995 [27]	86	IV	13	10.1	12	Age, volume
Larson et al., 1996 [31]	93	IV	16	6.5	16.4	Age, grade, KPS, focality, and volume
Kondziolka et al., 1997 [36]	42	III–IV	15.5	6.5	21	Grade, volume
Cho et al., 1999 [23]	46	III–IV	17	10	11	Age, grade, KPS, and volume
Ulm et al., 2005 [30]	33	III–IV	15	—	—	Location, RPA
Hsieh et al., 2005 [24]	26	IV	12	21.6	10	KPS
Mahajan et al., 2005 [37]	41	IV	—	4.7	11	None
Combs et al., 2005 [21]	32	IV	15	10	10	None
Kong et al., 2008 [13]	114	III–IV	16	10.6	26 (III)–13 (IV)	Histology, volume
Patel et al., 2009 [18]	26	IV	18	10.4	8.5	None
Biswas et al., 2009 [38]	18	IV	15	8.4	5.3	NR
Villavicencio et al., 2009 [25]	26	IV	20	7	7	Extent of surgery
Pouratian et al., 2009 [22]	26	IV	6	21.3	9.4	KPS, PTV margin
Torok et al., 2011 [39]	14	IV	24	6.97	10	NR
Maranzano et al., 2011 [40]	13	IV	17.3	5.3	11	Radiation dose
Cuneo et al., 2012 [29]	63	III/IV	15	4.8	11	Age, KPS, and bevacizumab
Park et al., 2012 [41]	11	IV	16	13.6	17.9	None
Skeie et al., 2012 [17]	51	IV	12.2	12.4	19 (from initial diagnosis)	None
Martínez-Carrillo 2014	87	III/IV	18.01	8.7	10 (17 III–7.5 IV)	KPS, RPA, histology, and PTV margin

NR: not reported.
